The article "Network Architecture for Optimizing Deep Deterministic Policy Gradient Algorithms" was published in 2022. Journal: Comput Intell Neurosci.

# Network Architecture for Optimizing Deep Deterministic Policy Gradient Algorithms

**DOI:** 10.1155/2022/1117781

**Published:** 2022-11-18

**Authors:** Haifei Zhang, Jian Xu, Jian Zhang, Quan Liu

**Affiliations:** ^1^School of Computer and Information Engineering, Nantong Institute of Technology, Yongxing Road 211, Nantong 226002, China; ^2^School of Information Science and Technology, Nantong University, Seyuan Road 9, Nantong 226019, China; ^3^School of Computer Science and Technology, Soochow University, Shizi Street 1, Suzhou 215006, China

## Abstract

The traditional Deep Deterministic Policy Gradient (DDPG) algorithm has been widely used in continuous action spaces, but it still suffers from the problems of easily falling into local optima and large error fluctuations. Aiming at these deficiencies, this paper proposes a dual-actor-dual-critic DDPG algorithm (DN-DDPG). First, on the basis of the original actor-critic network architecture of the algorithm, a critic network is added to assist the training, and the smallest *Q* value of the two critic networks is taken as the estimated value of the action in each update. Reduce the probability of local optimal phenomenon; then, introduce the idea of dual-actor network to alleviate the underestimation of value generated by dual-evaluator network, and select the action with the greatest value in the two-actor networks to update to stabilize the training of the algorithm process. Finally, the improved method is validated on four continuous action tasks provided by MuJoCo, and the results show that the improved method can reduce the fluctuation range of error and improve the cumulative return compared with the classical algorithm.

## 1. Introduction

As artificial intelligence continues to thrive, reinforcement learning (RL), which is a learning process that combines exploration and action, has been well developed in discrete action spaces focusing on decision control. By letting the agents learn continuously in a way of trial and error, RL pursues the overall maximum return while seeking the optimal action policy [1, 2]. However, when high-dimensional inputs or continuous action tasks are involved, traditional RL that relies on maximizing expected returns by performing trial and error may not work well. To tackle these kinds of problems, the concept of deep reinforcement learning (DRL) has been presented. In 2013, DeepMind proposed a method of using deep neural networks to play Atari games. It is the first successful and versatile DRL algorithm, although its scope of application is still limited to low-dimensional discrete action spaces. The topics dealing with continuous action tasks have become a new set of research interests [3, 4].

The article "Network Architecture for Optimizing Deep Deterministic Policy Gradient Algorithms" was published in 2022. Journal: Comput Intell Neurosci.

The basic idea of deep reinforcement learning is to fit the value function and policy function in reinforcement learning through a neural network. Typical algorithms include Deep *Q*-Network (DQN) [5] based on discrete action tasks and Deep Deterministic Policy Gradients (DDPG) [6] based on continuous action tasks. DDPG and DQN have very high similarities in algorithms. The main difference is that DDPG introduces a policy network to output continuous action values. DDPG can be understood as an extension algorithm of DQN in continuous action. DDPG algorithm has been studied extensively with a series of outcomes obtained. Mnih et al. [7] proposed the concept of two-layer BP neural network and hence improved the DDPG algorithm. The search efficiency of BP network was improved by using Armijo-Goldstein-based criterion and BFGS method [8]. Nikishin et al. [9] reduced the influence of noise on the gradient by averaging methods under the premise of random weights. Parallel actor networks and prioritized experience replay are used and tested in the continuous action space of bipedal robots [10]. The experimental results show that the revised algorithm can effectively improve the training speed. In addition, the storage structure of experience in DDPG is optimized, which improves the convergence speed of the DDPG algorithm through binary tree [11–13].

To sum up, the above methods propose improvements to address the shortcomings of DDPG, and all have achieved good results. Although the performance of the improved algorithms has been significantly improved, the flaws of local optimal solutions and large error fluctuations need to be further addressed.

The main content of this paper is as follows: Firstly, the basic principle of DDPG is introduced, and then, combined with the description of the network structure and its associated parameters, the existing shortcomings are also analyzed. Secondly, an improved algorithm is proposed to tackle the shortcomings of DDPG. The improvement method is mainly divided into two aspects. First, in order to reduce the probability of local optimal solutions, a critic network is added to assist training, and the smallest *Q* value in the two critic networks is taken as the estimated value of the action. Second, the dual-critic network will select the suboptimal *Q* value to update each round, and the suboptimal *Q* value also corresponds to the suboptimal action, which leads to the continuous underestimation of the action value of the agent. In response to this problem, this work introduces a dual-actor network based on the dual-critic network architecture; that is, the most valuable action in the two action networks is selected for training under the minimum *Q* value, so as to improve the robustness of the network structure. Finally, the effectiveness of the improved method is verified in eight simulated, experimental environments.

The article "Network Architecture for Optimizing Deep Deterministic Policy Gradient Algorithms" was published in 2022. Journal: Comput Intell Neurosci.

The rest of this paper is organized as follows: The basics of DDPG are introduced in Section 2. In Section 3, the idea of improving the algorithm is elaborated.  Section 4 includes experimental results and analysis.  Section 5 summarizes the work and refers to the future works.

## 2. Deep Deterministic Policy Gradients

The problem that reinforcement learning needs to solve is how to let the agent learn what actions to take in an environment, so as to obtain the maximum sum of reward values [12–14]. The reward value is generally associated with the task goal defined by the agent. The DDPG algorithm is used to solve the reinforcement learning problem in continuous action space [6, 15–17]. The main process is as follows: Firstly, the experience data generated by the interaction between the agent and the environment is stored in the experience recall mechanism. Secondly, the sampled data is learned and updated through the actor-critic architecture, and finally the optimal policy is obtained. The structure of the DDPG algorithm is shown in Figure 1 [15].

Based on the deterministic policy gradient, the DDPG algorithm uses a neural network to simulate the policy function and the *Q* function and combines the deep learning method to complete the task training [16]. The DDPG algorithm continues with the organizational structure of the DQN algorithm and uses actor-critic as the basic architecture of the algorithm [17]. The combination of the concepts of the online network and the target network in the DQN algorithm with the actor-critic method makes both actor and critic modules in the DDPG have access to the structure of the online network and the target network [6, 18, 19].

During the training process, the agent in the current state S decides the action A that needs to be performed through the current actor network and then calculates the *Q* value of the current action and the expected return value *y*_*i*_=*R*+*γQ*′ according to the current critic network. Then, the actor target network selects the optimal action *A*′ among the actions that can be performed according to the previous learning experience, and the *Q*′ value of the future action is calculated by the critic target network. The parameters of the target network are periodically updated by the online network parameters of the corresponding module.

DDPG adopts a “soft” method to update the target network parameters; that is, the magnitude of each update of the network parameters is very small, which improves the stability of the training process [20–22]. The update coefficient is denoted as *τ*, then the “soft” update method can be expressed as

(1) $$\begin{array}{c} w^{\prime }=\tau w+\left(1-\tau \right)w^{\prime }\theta^{\prime }=\tau \theta +\left(1-\tau \right)\theta^{\prime }\text{.} \end{array}$$

DDPG makes the decision of using action *a*_*t*_ by the deterministic policy *π*. It approximates the state-action function via a value network, with the definition of the target function as the accumulated reward with a discounted factor [23, 24] as shown in the following equation:

(2) $$\begin{array}{c} J\left(\theta \right)=E_{\theta }\left[r_{1}+{\gamma r}_{2}+\gamma^{2}r_{3}+\ldots \right]\text{.} \end{array}$$

In the online network of the critic, the update of the network parameters is based on the minimal value of the mean square error of the loss function [10], which can be expressed as

(3) $$\begin{array}{c} J\left(w\right)=\frac{1}{m}\overset{m}{\underset{j=1}{\sum }}\left(y_{j}-Q\left(ø\left(S_{j}\right),A_{j},w\right)\right){}^{2}\text{.} \end{array}$$

For the actor online network, the network parameters are updated according to the loss gradients of the policy [10] as shown in the following equation:.

(4) $$\begin{array}{c} \nabla_{J}\left(\theta \right)=\frac{1}{m}\overset{m}{\underset{j=1}{\sum }}\left[\nabla_{a}Q\left(s_{j},a_{j},w\right)|\nabla_{\theta_{\pi }}\right]\text{.} \end{array}$$

The article "Network Architecture for Optimizing Deep Deterministic Policy Gradient Algorithms" was published in 2022. Journal: Comput Intell Neurosci.

## 3. The DDPG Based on Dual-Actors and Dual-Critics

### 3.1. Error Analysis

It is an inevitable problem for *Q*-Learning to tend to overestimate errors [25–28]. In *Q*-Learning, the update of the estimated value of an action by the learning algorithm is conducted by the *ε*-greedy policy *y*_*t*_=*r*+*γ* max (*Q*(*s*_*t*+1_, *a*_*t*+1_)), hence the actual maximal value of an action is usually smaller than the estimated maximal value of this action as shown in the following equation:

(5) $$\begin{array}{c} E_{\epsilon }\left[\max_{a^{\prime }}\left(Q\left(S^{\prime },a^{\prime }\right)+\epsilon \right)\right]\geq \max_{a^{\prime }}Q\left(S^{\prime },a^{\prime }\right)\text{.} \end{array}$$

Equation (5) has already been proved for its establishment [29, 30]. Even the zero mean error of the initial state will lead to an overestimation of the action value due to the update of the value function, and the adverse effect of this error will be gradually enlarged by the calculation of the Bellman equation.

In the structure of actor-critic, the update of the actor policy depends on the critic value function [31–33]. Given the online network parameter *φ*, *ϕ*_approx_ denotes the updated parameter of the actor network calculated by the estimated maximal value function max (*Q*_*θ*_(*s*, *a*)), *ϕ*_true_ denotes the parameter obtained by using the actual value function *Q*_*π*_(*s*, *a*), where *Q*_*π*_(*s*, *a*) is unknown in the training process which represents the value function in an ideal state, then *ϕ*_approx_ and *ϕ*_true_ can be expressed in the following equation:

(6) $$\begin{array}{c} \phi_{approx}=\phi +\frac{\alpha }{Z_{1}}E_{s∼p_{\pi }}\left[{\nabla_{\phi }\pi_{\phi }\left(s\right)\nabla_{a}Q_{\theta }\left.s,a\right|}_{a=\pi_{\phi }\left(s\right)}\right]\text{,}\\ \phi_{true}=\phi +\frac{\alpha }{Z_{2}}E_{s∼p_{\pi }}\left[{\nabla_{\phi }\pi_{\phi }\left(s\right)\nabla_{a}Q^{\pi }\left.s,a\right|}_{a=\pi_{\phi }\left(s\right)}\right]\text{.} \end{array}$$

In Equation (6), *Z*_1,2_^−1^||*Е*[*·*]||=1, which normalizes gradients by using *Z*_1_ and *Z*_2_. Otherwise, highly estimated errors would have been a certain case in a strict constraint if gradient normalization had not been used [34, 35].

The article "Network Architecture for Optimizing Deep Deterministic Policy Gradient Algorithms" was published in 2022. Journal: Comput Intell Neurosci.

Since the gradient is updated in the direction of the local maximum, there is a very small number *k*1, so that when the learning rate of the neural network is less than *k*1. The parameter *π*_approx_ based on *ϕ*_approx_ and the parameter *π*_true_ based on *ϕ*_true_ converge to the local optimal value of the corresponding *Q* function, at this time, the estimation of *π*_approx_ is restricted to be below *π*_true_ as shown in the following equation:

(7) $$\begin{array}{c} \begin{array}{c} E\left[Q_{\theta }\left(s,\pi_{approx\;}\left(s\right)\right)\right]\geq E\left[Q_{\theta }\left(s,\pi_{true\;}\left(s\right)\right)\right]\text{.} \end{array} \end{array}$$

On the contrary, there is an extremely small number *k*2, so that when the learning rate of the neural network is less than *k*2, the parameter *π*_approx_ and the parameter *π*_true_ also converge to the local optimal value of the corresponding *Q* function, and the estimation of *π*_true_ is limited below *π*_approx_.

(8) $$\begin{array}{c} \begin{array}{c} E\left[Q_{\theta }\left(s,\pi_{true\;}\left(s\right)\right)\right]\geq E\left[Q_{\pi }\left(s,\pi_{approx\;}\left(s\right)\right)\right]\text{.} \end{array} \end{array}$$

If the training effect of the critic network is satisfying, the estimation of the policy value will be at least similar to the actual value of *φ*_true_ as shown in the following equation:

(9) $$\begin{array}{c} \begin{array}{c} E\left[Q_{\theta }\left(s,\pi_{true\;}\left(s\right)\right)\right]\geq E\left[Q_{\pi }\left(s,\pi_{true\;}\left(s\right)\right)\right]\text{.} \end{array} \end{array}$$

At this time, if the learning rate of the network is smaller than the smaller one of *k*1 and *k*2, we know by combining Equations (8) and (9), the action value will be overestimated as shown in the following equation:

(10) $$\begin{array}{c} \begin{array}{c} E\left[Q_{\theta }\left(s,\pi_{approx\;}\left(s\right)\right)\right]\geq E\left[Q_{\pi }\left(s,\pi_{approx\;}\left(s\right)\right)\right]\text{.} \end{array} \end{array}$$

The existence of errors will lead to inaccurate estimation of the action value, making the suboptimal policy be taken as the optimal policy output of the online network, thereby affecting the performance of the algorithm.

The article "Network Architecture for Optimizing Deep Deterministic Policy Gradient Algorithms" was published in 2022. Journal: Comput Intell Neurosci.

### 3.2. Dual-Actors and Dual-Critics Network Structure

Due to the existence of the overestimated error, the estimation of the value function can be used as an approximate upper limit of the estimated value of the future state. If there is a certain error in every *Q* value update, the accumulation of errors will result in a suboptimal policy. Aiming at this kind of problem, an additional critic network is used in this work. The smallest *Q* value of the two networks is taken as the estimated value of the action in each update, so as to reduce the adverse effect of the overestimated error.

The process of obtaining the smallest *Q* value via the dual-critic network is shown in the following equation:

(11) $$\begin{array}{c} y_{1}=r_{t+1}+\gamma Q_{1}^{\prime }\left(s_{t+1},\mu^{\prime }\left(s_{t+1}|\theta^{\mu^{\prime }}\right)\right)y_{2}=r_{t+1}+\gamma Q_{2}^{\prime }\left(s_{t+1},\mu^{\prime }\left(s_{t+1}|\theta^{\mu^{\prime }}\right)\right)y=\min\;\left(y_{1},y_{2}\right)\text{.} \end{array}$$

Although the dual-critic network can reduce the overestimated error of the algorithm and reduce the probability of generating a local optimal strategy, in the actual training process, it is rare for the learning rate of the neural network to be less than the minimum value of *k*1 and *k*2. Combined with Section 3.1 analysis, that is, the probability of overestimation is very low. The dual-critic network will select the suboptimal *Q* value to update in each round. The suboptimal *Q* value also corresponds to the suboptimal action, which leads to the continuous underestimation of the action value of the agent, and in turn affects the rate of convergence of the critic network [36–38].

Aiming at the problem of underestimation of the dual-critic network, in this work a dual-actor network is presented for training on the basis of the dual-critic network architecture. The network selects the action with the highest value among the two actions under the minimum *Q* value, which is used to reduce the influence of the *Q* value underestimation and improve the robustness of the network structure.

The article "Network Architecture for Optimizing Deep Deterministic Policy Gradient Algorithms" was published in 2022. Journal: Comput Intell Neurosci.

The network structure of the dual-actors and dual-critics is shown in Figure 2.

For a two-actor network, the training of this network is subject to the same issues upon the use of the same sample data and processing methods. In order to ameliorate this kind of problems, the update of the parameters of the two-actor network is based on different policy gradients, which helps to reduce the coupling between the two-actors and further improves the convergence rate of the algorithm [39, 40].

If the policies of the two-actors are defined as *π*_1_ and *π*_2_, and the parameters of the dual-critic network are *θ*_1_ and *θ*_2_, we will have two actions a_1_ = *μ* (s| *π*_1_) and a_2_ = *μ* (s| *π*_2_), then we can select the action with the maximal value based on this dual-actor network by using the following equation:

(12) $$\begin{array}{c} a={argmax}_{a}\max\;\left[Q_{1}\left(s,\mu \left(\left.s\right|\pi_{1}\right);\theta_{1}\right),Q_{2}\left(s,\mu \left(s\rfloor \pi_{2}\right);\theta_{2}\right)\right]\text{.} \end{array}$$

### 3.3. Modeling the Algorithm

Combining the ideas proposed in Section 3.2, this paper proposes a dual-actor and dual-critics based DDPG algorithm (DN-DDPG). The process of the DN-DDPG algorithm is shown in Algorithm 1.

## 4. Experiments

### 4.1. Software and Hardware Setup

The software environment used in this work is Anaconda3 4.8.3 (Python 3.8), the integrated development environment (IDE) is Pycharm, TensorFlow-GPU 1.8.0 is used as the learning framework. Python virtual environment is run in Anaconda3. NVIDIA GeForce GTX 1650 + CUDA 11.1 is the hardware environment.

### 4.2. Experimental Setup

In this paper, the Arm environment is written based on the Pyglet module. Two classical controls on the OpenAI GYM [20] platform and four continuous control tasks in the Mujoco physics simulator [21] are used as the experimental environment. OpenAI GYM is an open source toolkit that provides a variety of game environment interfaces to facilitate the research and development of artificial intelligence experiments.

The Arm environment used in this work includes the following items:

1. Arm_easy. 400 *∗* 400 2-dimensional space is constructed in the Arm environment. One end of a robot arm is fixed in the middle of the environment. The goal of the training is to make the other end of the robot arm find the blue target point as shown in Figure 3.
2. Arm_hard. This is similar to the Arm_easy environment, the only difference is that the target point is randomly generated in each round.

Two classical, continuous control task used in this work are shown below.

1. Pendulum. The pendulum starts at a random position, the aim is to push it swing upwards and keep erected.
2. Mountain Car Continuous. This task is to drive a car to reach the top of a hill; however, the power of the car is not sufficient to drive it directly to reach the top, it needs to rise and drop on the left and right sides repeatedly so that it can accumulate power to reach the top. It is shown in Figure 4.

The article "Network Architecture for Optimizing Deep Deterministic Policy Gradient Algorithms" was published in 2022. Journal: Comput Intell Neurosci.

The 4 Mujoco continuous control tasks include:

1. Half Cheetah. Train a bipedal agent to learn running as shown in Figure 5.
2. Hopper. Train a single legged robot to learn jumping forward.
3. Humanoid. Train a 3-dimensional bipedal agent to learn standing without falling down.
4. Walker2d. Train a 3-dimensional bipedal agent to walk forward as fast as possible.

This work compares the performance of DN-DDPG and the original DDPG algorithm. In order to study the improvement effect of the dual-critic network and the dual-actor network, the DCN-DDPG algorithm which is the single-actor and dual-critic network is included for comparison. The outcomes of the comparison are shown intuitively through experiments.

### 4.3. Parameter Setting

To ensure the accuracy and fairness of the experimental results, the common parameter values of different algorithms are the same. The training rounds for both the Arm environment and the two Gym classic control tasks are set to 2000 times, and the maximum number of training steps per round is 300 times. The training rounds of 4 kinds of Mujoco continuous control tasks are set to 5000 times, and the number of training steps per round is the maximum number of round steps in the Gym environment. The agent continuously learns and explores in the environment. If the preset task in the environment is successfully completed or the number of training times per round exceeds the maximum number of times, the scene will be reset and a new round will be started. Some parameters in the MuJoCo task are shown in Table 1.

### 4.4. Experimental Outcomes

In this work, the performances of three algorithms, DN-DDPG, DCN-DDPG and original DDPG, are compared in terms of their performance in two Arm environments, two Gym classical control environments, and four continuous tasks in Mujoco. DN-DDPG and DCN-DDPG are both based on the improvement of the DDPG method, the difference is that DCN-DDPG is based on the original DDPG with addition of an extra critic network, while DN-DDPG is based on the DCN-DDPG with addition of an extra actor network to optimizing training. The comparison of these three algorithms can make a more intuitive display of the two improved methods mentioned in this article: dual-critics and dual-actors. The experimental results are shown in Figure 6.

The shaded part in the figure represents the standard deviation during training, that is, when using the same hyperparameters and network model, different random number seeds are used to achieve random exploration. The shaded upper limit is the optimal result. The *x*-axis represents the number of rounds of agent training, the *y*-axis represents the cumulative reward obtained per round, and the experiment recorded the average reward value per 100 rounds.

The article "Network Architecture for Optimizing Deep Deterministic Policy Gradient Algorithms" was published in 2022. Journal: Comput Intell Neurosci.

In the environments of Arm easy and Arm hard, the average rewards from three algorithms stay around a same value. In some cases, the rewards from both DCN-DDPG and DDPG are superior to that of DN-DDPG. However, from the point of view of overall training effects, DN-DDPG performs better than the other two algorithms, while DCN-DDPG is slightly better than DDPG. In Pendulum experiment, the overall performance of the DN-DDPG is the best, which is due largely to the fact that dual-critics network is able to reduce the error while dual-actors network selects the action of higher value. In cases of Mountain Car Continuous, the average rewards from these three algorithms tend to be the same. However, during the process of 200 time steps, DN-DDPG has a better convergence speed than the rest two algorithms. In addition, in Half Cheetah, Humanoid, Hopper and Walker2d, DN-DDPG has a worse starting performance than DCN-DDPG and DDPG, which could be due to the fact that DCN-DDPG and DDPG have relatively simpler network structure able to deal with complex environment easier than DN-DDPG. The DN-DDPG needs a period for training, and after this initial training period the average reward from DN-DDPG becomes obviously better than the rest two algorithms. Again, the overall performance of DCN-DDPG is better than DDPG. Finally, the shaded areas of different algorithms are compared, with the outcomes that the area of DN-DDPG is smaller than those of DCN-DDPG and DDPG, which reflects that the training of DN-DDPG is more stable.

From the experimental results in Figure 6, the dual-critics method is able to increase the performance of DDPG algorithm, but to a limited extent. By introducing dual-actors method, the DN-DDPG network, based on the DCN-DDPG, is able to further increase the overall performance and training stability of the algorithm. Hence, compared to the original DDPG, the DN-DDPG which is based on dual-actors and dual-critics, has the best increased performance.

## 5. Conclusion

A deep deterministic policy gradient algorithm is proposed based on a dual-actors and dual-critics network. In order to reduce the overestimated error in the original actor-critic network, a dual-critics target network is introduced into the algorithm, and the minimum action estimate generated by the two networks is selected to update the policy network. In order to alleviate the problem of underestimation caused by the dual-critics network, a dual-actors network is added on the basis of the original network, and the action with the highest value among the two actions generated by the dual-actors network is selected. The experimental results show that, compared with the original DDPG algorithm, and the DDPG algorithm based on the single-actor and two-critics network, the novel DN-DDPG algorithm based on the dual-actors and dual-critics network has a higher cumulative reward and a smaller standard deviation of training.

The article "Network Architecture for Optimizing Deep Deterministic Policy Gradient Algorithms" was published in 2022. Journal: Comput Intell Neurosci.

There is more to be explored in future work. First, in order to improve the optimization ability of the algorithm, more suitable deep learning methods can be explored and applied to neural networks. Second, for the experience replay mechanism in the DDPG algorithm, it is viable to explore whether there is a better method to determine the sample priority to improve the convergence speed during training.

## Figures and Tables

**Figure 1:** The structure of DDPG algorithm.

**Figure 2:** Architecture of dual-actors and dual-critics.

**Figure 3:** Arm_easy environment and task.

**Figure 4:** Mountain car continuous.

**Figure 5:** Half cheetah.

**Figure 6:** Comparative experiments of three algorithms in eight different continuous action tasks. (a) Arm_easy. (b) Arm_hard. (c) Pendulum. (d) Mountain car continuous. (e) Half cheetah. (f) Humanoid. (g) Hopper. (h) Walker2d.

**Algorithm 1:** The DN-DDPG process.

**Table 1:** Mujoco environment model hyperparameters.

Order	Parameter	Value
1	Decay rate	0.9
2	Actor net learning rate	0.0001
3	Critic net learning rate	0.0001
4	Neuron number in 1^st^ layer	400
5	Neuron number in 2^nd^ layer	300
6	Experience pool volume	100000
7	Batch data size	256
8	Soft update coefficient	0.01
9	Action reward discount rate	0.99
10	Critic net output distribution low limit	−20
11	Target net parameters update round number	10

## Data Availability

The dataset can be accessed upon request.

## References

[1] Dörpinghaus M., É R., Neri I., Meyr H., Jülicher F. An information theoretic analysis of sequential decision-making.

[2] Liu Q., Zhai J. W., Zhang Z.-Z., Zhong S., Zhou Q., Zhang P. (2018). A survey on deep reinforcement learning. *Chinese Journal of Computers*.

[3] Hasselt H. V., Wiering M. A. Using continuous action spaces to solve discrete problems.

[4] Zhang W., Chen Q., Yan J., Zhang S., Xu J. (2021). A novel asynchronous deep reinforcement learning model with adaptive early forecasting method and reward incentive mechanism for short-term load forecasting. *Energy*.

The article "Network Architecture for Optimizing Deep Deterministic Policy Gradient Algorithms" was published in 2022. Journal: Comput Intell Neurosci.

[5] Yang Y., Juntao L., Lingling P. (2020). Multi‐robot path planning based on a deep reinforcement learning DQN algorithm. *CAAI Transactions on Intelligence Technology*.

[6] Zhou Q. (2020). A novel movies recommendation algorithm based on reinforcement learning with DDPG policy. *International Journal of Intelligent Computing and Cybernetics*.

[7] Mnih V., Kavukcuoglu K., Silver D. (2013). Playing atari with deep reinforcement learning. https://arxiv.org/abs/1312.5602.

[8] Zhang M., Zhang Y., Gao Z., He X. (2020). An improved DDPG and its application based on the double-layer BP neural network. *IEEE Access*.

[9] Nikishin E., Izmailov P., Athiwaratkun B. Improving stability in deep reinforcement learning with weight averaging.

[10] Wu X., Liu S., Zhang T. Motion control for biped robot via DDPG-based deep reinforcement learning.

[11] Tang J., Li L., Ai Y. Improvement of End-To-End Automatic Driving Algorithm Based on Reinforcement Learning.

[12] Sutton R. S., Barto A. G. (2018). *Reinforcement Learning: An Introduction*.

[13] Zhang Y., Zhao B., Liu D. (2020). Deterministic policy gradient adaptive dynamic programming for model-free optimal control. *Neurocomputing*.

[14] Chu Y., Fei J., Hou S. (2020). Adaptive global sliding-mode control for dynamic systems using double hidden layer recurrent neural network structure. *IEEE Transactions on Neural Networks and Learning Systems*.

[15] Zhang H., Xu J., Lei L. (2021). *A Manipulator Control Method Based on Deep Deterministic Policy Gradient with Parameter Noise*.

[16] Liu J., Gao F., Luo X. (2019). Survey of deep reinforcement learning based on value function and policy gradient. *Chinese Journal of Computers*.

[17] Mizutani E., Dreyfus S. (2017). Totally model-free actor-critic recurrent neural-network reinforcement learning in non-Markovian domains. *Annals of Operations Research*.

[18] Xiang Y., Wen J., Luo W., Xie G. Research on collision-free control and simulation of single-agent based on an improved DDPG algorithm.

[19] Thrun S., Schwartz A. Issues in using function approximation for reinforcement learning.

[20] Brockman G., Cheung V., Pettersson L. (2016). OpenAI gym. CORR. https://arxiv.org/abs/1606.01540.

[21] Todorov E., Erez T., MuJoCo Y. T. A physics engine for model-based control.

[22] Fu X., Zhu J., Wei Z., Wang H., Li S. (2022). A UAV pursuit-evasion strategy based on DDPG and imitation learning. *International Journal of Aerospace Engineering*.

[23] Li L., Hang J., Sun H., Wang L. (2017). A conjunctive multiple-criteria decision-making approach for cloud service supplier selection of manufacturing enterprise. *Advances in Mechanical Engineering*.

The article "Network Architecture for Optimizing Deep Deterministic Policy Gradient Algorithms" was published in 2022. Journal: Comput Intell Neurosci.

[24] Li L. h, Hang J. c, Gao Y., Mu C. Y. (2017). Using an integrated group decision method based on SVM, TFN-RS-AHP, and TOPSIS-CD for cloud service supplier selection. *Mathematical Problems in Engineering*.

[25] Li P., Ding X., Sun H., Zhao S., Cajo R. (2021). Research on dynamic path planning of mobile robot based on improved DDPG algorithm. *Mobile Information Systems*.

[26] Li L., Lei B., Mao C. (2022). Digital twin in smart manufacturing. *Journal of Industrial Information Integration*.

[27] Li L., Mao C., Sun H., YuanLei B. (2020). Digital twin driven green performance evaluation methodology of intelligent manufacturing: hybrid model based on fuzzy rough-sets AHP, multistage weight synthesis, and PROMETHEE II. *Complexity*.

[28] Du Y., Zhang X., Cao Z. (2021). An optimized path planning method for coastal ships based on improved DDPG and DP. *Journal of Advanced Transportation*.

[29] Yao Z., Wang Y., Meng L., Qiu X., Yu P. (2021). DDPG-based energy-efficient flow scheduling algorithm in software-defined data centers. *Wireless Communications and Mobile Computing*.

[30] Wu R., Gu F., Liu H.-L., Shi H. (2022). UAV path planning based on multicritic-delayed deep deterministic policy gradient. *Wireless Communications and Mobile Computing*.

[31] Zhang L., Pan Z., Pan Yu (2022). A hidden attack sequences detection method based on dynamic reward deep deterministic policy gradient. *Security and Communication Networks*.

[32] Li Y., Li L. H. (2020). Enhancing the optimization of the selection of a product service system scheme: a digital twin-driven framework. *Strojniški vestnik - Journal of Mechanical Engineering*.

[33] Li L. H., Wang H. G. (May 16 2018). A VVWBO-BVO-based GM (1, 1) and its parameter optimization by GRA-IGSA integration algorithm for annual power load forecasting. *PLoS One*.

[34] Zhang H., Xu J., Qiu J. (2022). An automatic driving control method based on deep deterministic policy gradient. *Wireless Communications and Mobile Computing*.

[35] Yuan W., Xiwen Z., Rong Z., Shangqin T., Huan Z., Wei D. (2022). Research on UCAV maneuvering decision method based on heuristic reinforcement learning. *Computational Intelligence and Neuroscience*.

[36] Chen J., Wang Y., Ou J. (2022). ALBRL: automatic load-balancing architecture based on reinforcement learning in software-defined networking. *Wireless Communications and Mobile Computing*.

[37] Li L., Qu T., Liu Y., ZhongXuSunGaoLeiMaoPanWangMa C. (2020). Sustainability assessment of intelligent manufacturing supported by digital twin. *IEEE Access*.

[38] Li L., Mao C. (2020). Big data supported PSS evaluation decision in service-oriented manufacturing. *IEEE Access*.

The article "Network Architecture for Optimizing Deep Deterministic Policy Gradient Algorithms" was published in 2022. Journal: Comput Intell Neurosci.

[39] Wang Zi-J., Chen X.-M., Wang P., Li M.-Xi, Ou Y.-J.-X., Zhang H. (2021). A Decision-making model for autonomous vehicles at urban intersections based on conflict resolution. *Journal of Advanced Transportation*.

[40] Chen Xi-L., Cao L., Xu Z.-X., Lai J., Li C.-Xi (2019). A study of continuous maximum entropy deep inverse reinforcement learning. *Mathematical Problems in Engineering*.

